The article "Brain Tumor Detection and Classification by MRI Using Biologically Inspired Orthogonal Wavelet Transform and Deep Learning Techniques" was retracted in 2023. Reasons: unreliable results or conclusions; concerns about the data; concerns about the peer review; concerns about the citations.

# Brain Tumor Detection and Classification by MRI Using Biologically Inspired Orthogonal Wavelet Transform and Deep Learning Techniques

**DOI:** 10.1155/2022/2693621

**Published:** 2022-01-10

**Authors:** Muhammad Arif, F. Ajesh, Shermin Shamsudheen, Oana Geman, Diana Izdrui, Dragos Vicoveanu

**Affiliations:** ^1^Department of Computer Science and Information Technology, University of Lahore, Lahore, Pakistan; ^2^Department of Computer Science and Engineering, Sree Buddha College of Engineering, Alappuzha, Kerala, India; ^3^College of Computer Science and Information Technology, Jazan University, Jazan, Saudi Arabia; ^4^Neuroaesthetics Lab, Stefan cel Mare University of Suceava, Suceava, Romania; ^5^Faculty of Electrical Engineering and Computer Science, Stefan cel Mare University of Suceava, Suceava, Romania

## Abstract

Radiology is a broad subject that needs more knowledge and understanding of medical science to identify tumors accurately. The need for a tumor detection program, thus, overcomes the lack of qualified radiologists. Using magnetic resonance imaging, biomedical image processing makes it easier to detect and locate brain tumors. In this study, a segmentation and detection method for brain tumors was developed using images from the MRI sequence as an input image to identify the tumor area. This process is difficult due to the wide variety of tumor tissues in the presence of different patients, and, in most cases, the similarity within normal tissues makes the task difficult. The main goal is to classify the brain in the presence of a brain tumor or a healthy brain. The proposed system has been researched based on Berkeley's wavelet transformation (BWT) and deep learning classifier to improve performance and simplify the process of medical image segmentation. Significant features are extracted from each segmented tissue using the gray-level-co-occurrence matrix (GLCM) method, followed by a feature optimization using a genetic algorithm. The innovative final result of the approach implemented was assessed based on accuracy, sensitivity, specificity, coefficient of dice, Jaccard's coefficient, spatial overlap, AVME, and FoM.

## 1. Introduction

Every year, more than 190,000 people in the world are diagnosed with primary or metastatic brain (secondary) tumors. Although the causes of brain tumors are not certain, there are many trends among the people who get them. Any human being, whether a child or an adult, may be affected by it. The tumor region has initially identified a reduction in the risk of mortality [1]. As a result, the radiology department has gained prominence in the study of brain tumors using imaging methods. Many studies have looked at the causes of brain tumors, but the results have not been conclusive. In [2], an effective partitioning strategy was presented using the *k*-means clustering method integrated with the FCM technique. This approach will benefit from the *k*-means clustering in terms of the minimum time of calculation FCM helps to increase accuracy. Amato et al. [3] structured PC-assisted recognition using mathematical morphological reconstruction (MMR) for the initial analysis of brain tumors. Test results show the high accuracy of the segmented images while significantly reducing the time of calculation. In [4], classification of neural deep learning systems was proposed for the identification of brain tumors. Discrete wavelet transformation (DWT), excellent extraction method, and main component analysis (PCA) were applied to the classifier here, and performance evaluation was highly acceptable across all performance measurements.

In [5], a new classifier system was developed for brain tumor detection. The proposed system achieved 92.31% of accuracy. In [6], a method was suggested for classifying the brain MRI images using an advanced machine learning approach and brain structure analytics. To identify the separated brain regions, this technique provides greater accuracy and to find the ROI of the affected area. Researchers in [7] proposed a strategy to recognize MR brain tumors using a hybrid approach incorporating DWT transform for feature extraction, a genetic algorithm to reduce the number of features, and to support the classification of brain tumors by vector machine (SVM) [8]. The results of this study show that the hybrid strategy offers better output in a similar sense and that the RMS error is state-of-the-art. Specific segmentation concepts [9–33] include region-based segmentation [10], edge-based technique [11], and thresholding technique [12] for the detection of cancer cells from normal cells. Common classification method is based on the Neural Network Classifier [13], SVM Classifier [14], and Decision Classifier [15]. In [32], a brain tumor detection method was developed using the GMDSWS-MEC model. The result shows high accuracy and less time to detect tumors.

### 1.1. Research Gap Identified

From the research analysis, we have identified that traditional algorithms are very effective to the initial cluster size and cluster centers. If these clusters vary with different initial inputs, then it creates problems in classifying pixels. In the existing popular fuzzy cluster mean algorithm, the cluster centroid value is taken randomly. This will increase the time to get the desired solution. Manual segmentation and evaluation of MRI brain images carried out by radiologists are tedious; the segmentation is done by using machine learning techniques whose accuracy and computation speed are less. Many neural network algorithms have been used for the classification and detection of the tumor where the accuracy is less. The detection accuracy is based on the segmentation and the detection algorithms used. So far, in an existing system, the accuracy and the quality of the image are less.

### 1.2. Contribution of the Proposed Research

The proposed technique is an effective technique to detect tumour from MRI images. In the proposed technique, different classifiers are used. The proposed system should be capable of processing MRI, multislice sequences, accurately bounding the tumor area from the preprocessed image via skull stripping and morphological operations. The region should be segmented by Berkeley's wavelet transformation and extract the texture features using ABCD, FOS, and GLCM features. Classifiers such as Naïve Bayes, SVM-based BoVW, and CNN algorithm should compare the classified result and must identify the tumor region with high precision and accuracy. Finally, based on the classifier result, the tumor region is classified into malignant or benign.

The rest of the article is intended to continue: section 1 presents the background to brain tumors and related work; section 2 presents the construction techniques with the measures used throughout the method used; section 3 describes the results and analysis and the comparative study; and, finally, section 4 presents the conclusions and upcoming work.

## 2. Methodology

In this research work, the initial image database is collected; the obtained images are enhanced by thresholding, morphological operation, and region filling. After preprocessing, the tumor region is segmented using the BWT algorithm. The features are extracted by using the GLCM algorithm. The genetic algorithm is used for selecting the features. Finally, the SVM Naïve Bayes, BOV-based SVM classifier, and CNN classify the image accurately. The flow for identifying the brain tumors is portrayed in Figure 1.

### 2.1. Data Acquisition

The data collected are grouped into two kinds—healthy brain images and unhealthy brain images. Among the 66 patients, 22 patients have normal MRI brain images and the rest 44 collect in the abnormal MRI brain image category from the Harvard Medical School website (http://med.harvard.edu/AANLIB/) [16]. The MRI brain image obtained from the database were in the form of an axial plane, T2-weighted, and 256 × 256 pixels. These images are scrutinized, and preprocessing is done before the processing of algorithms.

### 2.2. Preprocessing

The preprocessing step focuses on specifically removing the redundancy present in the captured image without affecting the subtleties that play a key role in the general procedure. It is done to improve the visual look and characteristics of an image. In the conventional model, MRI images [34] are often affected by impulse noise, such as salt and pepper, which degrades the performance of the tumor segmentation system to avoid the proposed skull stripping and morphological operations.

The key activities in preprocessing are thresholding, morphological operation, and region filling. In the input image, at first, mean is calculated, and thresholding operation is done. To remove holes from the input image, region filling operation is done, which is trailed by morphological activity, with the goal that it can eliminate noise as well as small objects from the background. Normally, preprocessing can be assessed visually or quantitatively.

### 2.3. Segmentation-Berkeley's Wavelet Transformation

Segmentation is used to identify the tumor infected area from the MR images. The Berkeley wavelet transformation uses two-dimensional triadic wavelet transformation and a complete, orthonormal basis, and hence it is very ideal for the identification of the area of interest from the MR images [17]. The BWT converges repetitively from one level to *n*—number of levels—and decomposes the other part of the image at a very fast rate.

The partition of the highly contagious MR brain areas is done as follows:

- In the initial stage, the enhanced brain MRI image is transformed into a binary image with a cut-off level of 117. Pixels with values larger than the defined level are converted to white, whereas the remaining pixels are marked as black, resulting in the development of two distinct regions around the infected tumor tissues.
- In the second stage, the morphological erosion procedure is used to remove white pixels. Finally, the region is divided into destruction and identical areas, and the area of the omitted black pixels of the erosion process is counted as the MR image mask for the brain.

This present work deals with the conversion of Berkeley's wavelets, which is used to effectively section the brain MR image. The conversion of the Berkeley wavelet (BWT) is defined as the transformation of two-dimensional triadic wavelets, which can be used to analyze the signal or image. The BWT is used in features, such as spatial position, band pass frequency, band pass orientation tuning, quadrature phase, etc. As with the conversion of the mother wavelet or other wavelet transformation communities, the BWT algorithm will also allow for an efficient transition from one spatial form to a temporal domain frequency. The BWT is an important method of image transformation and is a complete orthonormal one.

BWT consists of eight major mother wavelets grouped into four pairs, each pair having different 0, 45, 90, and 135 degrees aspects. Inside each pair of wavelet transforms, some wavelet has odd symmetry, while another wavelet also has symmetry. The BWT algorithm is an accurate, orthonormal basis and is therefore useful for computational power reduction. Here, the Berkeley wavelet transformation is used for efficient division [18]. Wavelet analysis is an efficient approach capable of revealing data aspects which are other techniques for analyzing the signal. The process, by considering the images at numerous stages, can take out the finer details from them and in effect enhance the image quality. Alternatively, wavelet analysis can compress or denoise a signal without significant degradation. The BWT algorithm steps are defined as follows:

(1) Initially calculate scaling and translation process:
  (1) $$\begin{array}{c} P=\;\frac{1}{\sqrt{S}}\psi \left(\frac{T-\tau }{S}\right). \end{array}$$
(2) Perform conversion of data from a spatial form to a temporal domain frequency.
(3) Simplification of image conversion calculation of the mother wavelet transformation is partly fixed:
  (2) $$\begin{array}{c} \beta_{\theta }^{\phi }\left(\tau ,\;S\right)=\frac{1}{S^{2}}\beta_{\theta }^{\phi }\left(3^{S}\left(x-i\right),3^{S}\left(y-j\right)\right),\\ \beta_{0}=\frac{1}{\sqrt{9}}\left[\mu \left(\frac{x}{3},\frac{y}{3}\right)\right]. \end{array}$$
(4) Apply the morphological technique.
(5) Reschedule the corresponding pixel values; this process is only for binary images.
(6) Removing pixels from or to the edge area of the artifacts relies on just the streamlining element of the image selected.

### 2.4. Feature Extraction

The extraction procedure for the element is utilized to consequently find the lesion. There are three procedures to consider for the extraction of features: FOS, ABC, and GLCM.

#### 2.4.1. ABC Parameter

The extracted features based on ABC are given as follows:

(i) Asymmetry index:
  (3) $$\begin{array}{c} AI=\frac{A_{1}+A_{2}}{2A_{r}}. \end{array}$$
(ii) Four different border irregularity measures are
  (a) Compactness index:
    (4) $$\begin{array}{c} CI=\;\left(P2L\right)=\;4AL. \end{array}$$
  (b) Fractal index: The set of fractals is calculated using the tracking of boxes. The box tracking is portrayed by *N(S)* in the fractal dimension plot, and *N* symbolizes a sequence of boxes. Box track is described for the Hausdorff dimension plot with log *N(S)*, and log *N* signifies several columns.
  (c) Edge abruptness:
    (5) $$\begin{array}{c} \text{EI }=\frac{\left(\max.\min\right)\%6\;+\;2}{100}. \end{array}$$
  (d) Gray transition: It calculates the position and velocity of an image's gradient.
(iii) Diameter: The diameter of the lesion field is calculated for smaller axis length by using the function' region props' function. The resulting value is converted to a value of the nanometer, and that value is assigned the diameter.

#### 2.4.2. GLCM Features

This strategy obeys two measures to synthesize characteristics of the medicinal images. During the initial process, the GLCM features are computed and in the next process, the texture characteristics depending upon the GLCM are determined. The metric formula is depicted below for a few of the innovative features. Extraction of the feature is done using a co-occurrence matrix of the gray level [20]. Several texture features are available, but this study uses only four features: strength, contrast, correlation, and homogeneity.

(6) $$\begin{array}{c} \text{Energy}=\overset{G-1}{\underset{i=0}{\sum }}\overset{G-1}{\underset{j=0}{\sum }}{\left[p\left(x,y\right)\right]}^{2},\\ \text{Homogenity}=\;-\overset{G-1}{\underset{i=0}{\sum }}p\left(i\right)\log_{2}\left[p\left(x\right)\right],\\ \text{Correlation}=\overset{G-1}{\underset{i=0}{\sum }}\overset{G-1}{\underset{i=0}{\sum }}\frac{x,y\;p\left(x,y\right)-\;\mu_{x}\mu_{y}}{\sigma_{x}\sigma_{y}},\\ \text{Contrast}=\overset{G-1}{\underset{i=0}{\sum }}\overset{G-1}{\underset{j=0}{\sum }}\left(x-y\right)p\left(x,y\right). \end{array}$$

#### 2.4.3. Statistical Features

The descriptor Color Moment (CM) is used to derive both functions. Statistical Function Equations (FOS) are given below:

(7) $$\begin{array}{c} \text{Mean }\mu =\overset{G-1}{\underset{i=0}{\sum }}\text{i p}\left(x\right),\\ \text{Variance }\sigma^{2}=\;\overset{G-1}{\underset{i=0}{\sum }}{\left(x-\mu \right)}^{2}p\left(x\right),\\ \text{Skewness }\mu_{3}=\;\sigma^{-3}\overset{G-1}{\underset{i=0}{\sum }}{\left(x-\mu \right)}^{3}p\left(x\right),\\ \text{Kurtosis }\mu_{4}=\;\sigma^{-4}\overset{G-1}{\underset{i=0}{\sum }}{\left(x-\mu \right)}^{4}p\left(x\right),\\ \text{Entropy }H=-\;\overset{G-1}{\underset{i=0}{\sum }}\overset{G-1}{\underset{j=0}{\sum }}\;p\left(x,y\right)\log_{2}\left[p\left(x\right)\right]. \end{array}$$

Figure 2 shows 13 features that are selected for contributions to the classification system. The network consists of 4 hidden neurons, and 1 output neuron is used for the final examination of the network. At that point, the rules for choosing the component are utilized to diminish the quantity of feature input.

### 2.5. Features Selection Using Genetic Algorithm

Not all the features make a payment to the classification process. Feature selection is carried out to identify the most suitable feature set. We use the genetic algorithm to optimize the selected feature values for the proposed method because it offers significant advantages over typical optimization techniques, such as linear programming, heuristic, first depth, first breadth, and Praxis [21] Feature selection process is presented in Figure 3, and the procedure of GA is given in Algorithm 1.

#### 2.5.1. Features Selection: Genetic Algorithm

Genetic algorithms play an important role in reducing the dimensionality of the feature space, thus helping to improve the performance of the classifier. In the genetic algorithm, the major stages are fitness evaluation, chromosome encoding, selection technique, genetic operators, and the condition stops iteration. In binary search space, the genetic algorithm considers chromosomes to be a bit string.  Figure 4 shows the matrix representation showing the bit value of the chromosome in genetic algorithm.

Initially, a primary population is formed arbitrarily as well as by utilizing fitness function, it is assessed. In the testing, the chromosome with the bit string value “1” represents the specific feature indexed by the selected position. The ranking determines the accuracy of previously tested classification data. The chromosomes that have the highest fitness function are selected according to the ranking. The remaining chromosome has to undergo mutation and crossover to produce a greater likelihood of a new chromosome. This process is repeated until the attainment of a fitness function [22].

*(1) Initial Population Selection*. The initial population matrix is given by *m* × *n*, where *m* and *n* represent population size and chromosome length. In the present function, the number of derived features of the picture block is equal to the length of the chromosome, and the number of chromosomes indicates the size of the population. Each bit of a chromosome in the features matrix indicates the position of the feature. A “1” in the chromosome is the selection of the matrix of the equivalent feature.

#### 2.5.2. Fitness Evaluation

A fitness function has the original goal of assessing the discriminating capacity of each subset. Evaluating the reasonable number of the test data and the function space of the training sets solves the classification problem.

(8) $$\begin{array}{c} D\left(x_{test},x_{i}\right)=\sqrt{\overset{M}{\underset{m-1}{\sum }}{\left(x_{test}-x_{i}\right)}^{2}}. \end{array}$$

Since the GA iterates, dependent upon the classification error, the distinct chromosomes in the present population are assessed and the fitness is ranked as well. Iteration is mainly done to decrease the error rate and to find the smallest and best fitness value,

(9) $$\begin{array}{c} \text{fit}=\;\frac{\alpha }{N_{f}}+\text{Exp}\left(\frac{-1}{N_{f}}\right). \end{array}$$

Here, *N*_f_ = cardinality of the selected features and *α* = represents the classification error.

*(1) New Population for Generation of Children*. A new generation is established after evaluating the fitness function. It mainly depends on the genetic operator such as crossover and mutation. This new population is named: Elite, crossover, and mutation.

- *Elite Children*. Since these new populations are the finest children containing the highest fitness value, these are pushed automatically to the successive generation. The population size gives the total elite chromosome. This infers EliteCount ≤ populationSize.
- If the size of chromosomes is 2, the genetic algorithm chooses the two finest chromosomes and pushes them to the subsequent generation.
- *Crossover Children*. Crossover fraction is the ratio of the following generation besides the remaining kids, which are created by crossover. There are no children with mutations when the fraction is fixed to one.
- New Population: Mutation Children. Lastly, the number of mutation children is *M*_count_ = 100-EliteCount-COcount = 100-2-78 = 20. This infers Elite_Count_ + CO_count_ + *M*_count_ = 100.

*(2) Tournament*. In the genetic algorithm, the goal of the selection technique is to ensure the population is being persistently enhanced with complete fitness values. This technique aids the GA in eliminating poor designs as well as maintaining simply the finest individuals. There are a lot of selection techniques, for instance, stochastic uniform. In this proposed research, the selected tournament is having a size of 2 which is used because of its easiness, speed, and efficacy. Tournament selection always ensures in the selection process that the poorest individual does not go to the subsequent generation. To carry out tournament selection, two functions are required (i.e., the players (parents) and the winners). Two chromosomes of size 2 are selected in the tournament selection, from the elite children's population and finest of the two chromosomes. It is carried out iteratively by filling up a freshly produced population.

*(3) Crossover Function*. In the GA, to produce children for the next generation, the crossover operator genetically combines two individuals called parents. After the removal of elite kids, the number of new kids formed from the new population is given by the crossover kids and it is being evaluated. The crossover fraction normally has a value between 0 and 1. The present work crossover value is 0.8. Two-parent chromosomes have binary values and an XOR operation is carried out on these chromosomes.

### 2.6. Classification

Within the area of computers, vision classification is a significant chore. The labeling of images hooked on one of several defined groupings is called image classification. The classification scheme contains a database that holds predefined patterns that relates to the perceived item to organize into a suitable classification. Here, various techniques like Naïve Bayes, SVM-based BoVW, and CNN algorithm are used.

#### 2.6.1. Naïve Bayes Classifier

The classification of Naïve Bayes has played a major role in the extraction of medical data. It shows superior accuracy, performance because the attributes are independent of each other. The missing values arise continuously in the case of clinical data [35]. This naturally treats misplaced ideals as if lost by mistake. This algorithm replaces zeros with limited numerical data and zero vectors with categorical negative data. In nested columns, missing values are interpreted as being sparse. Missing values in columns with simple data types are interpreted as missing at random. Generally, when choosing to manage our data preparation, Naïve Bayes requires binning. It trusts to estimate the likelihood of accumulation of procedures [23]. To reduce the cardinality, the columns should be discarded as appropriate.

In principle, it has the base error rate in contrast with every other classifier. They give hypothetical avocation to different classifiers which do not expressly utilize the Naïve Bayes theorem. For example, it tends to be shown, based on specific presumptions, that numerous neural systems and curve-fitting calculations yield the most posterior hypothesis, as does the naïve Bayesian classifier. This classification is completed by using a probabilistic methodology that calculates the class probabilities and predicts the most likely classes. A Naïve Bayes classifier applies Bayesian statistics with strong, independent suspicions on the features that drive the classification procedure. It is the basic grouping conspires, which approximations the class conditional likelihood by expecting that the properties are restrictively autonomous, given the class name *c*. The conditional probability can be finally conveyed as pursues:

(10) $$\begin{array}{c} P\left(C|A\right)=c=\overset{n}{\underset{i=1}{\prod }}P\left(\frac{A_{i}}{C}\right)=c, \end{array}$$

wherever both attributes set *A* = {*A*1, *A*2 .... *An*} contains the capabilities of *n* attributes. With the restrictive probability ratio, instead of calculating the class conditional probability for each grouping of *A*, just estimate the conditional probability of each *A*_*i*_, given *C*. The last method is becoming increasingly useful as it does not entail an incredibly huge collection of preparations to get a reasonable estimate of the likelihood. Each classifier determines the posterior likelihood for each class *C* to be used to classify a test sample.

(11) $$\begin{array}{c} P\left(C|A\right)=\frac{P\left(C\right)\prod_{i=1}^{n}P\left(A_{i}/C\right)}{P\left(A\right)}. \end{array}$$

Since *P* (*A*) is fixed for each *A*, it is adequate to choose the class that boosts the numerator term:

(12) $$\begin{array}{c} P\left(C\right)\overset{n}{\underset{i=1}{\prod }}P\left(\frac{A_{i}}{C}\right). \end{array}$$

This classifier has a few benefits. It is informal to use different classification approaches; only one time scan of the training data is compulsory. The naïve Bayesian classifier can simply hold missing characteristic qualities by essentially precluding the probability when computing the probabilities of enrolment in each class.

#### 2.6.2. SVM Classification Based on BoV

BoVwords is a supervised model of learning and an extension to the NLP algorithm. Bag of Words is used for classification of images. It is used quite widely aside from CNN. In essence, BOV provides a vocabulary that can best describe the image in terms of extrapolating properties. By generating a bag of visual words, it uses the Computer Vision Toolbox^TM^ functions to define the image categories. The method produces histograms of occurrences of visual words; such histograms are used to classify the images. The steps of the support vector machine are presented in Figure 5.

The steps below explain how to set up your images, develop a bag of visual words, then train and apply a classifier for the image type [24].

It follows 4 simple steps:

- Ability of Image features of a defined label
- Development of visual vocabulary by clustering, accompanied by frequency analysis
- Classification of generating vocabulary-based images
- Obtain the best class for the query image.

The algorithm for the bag of visual classifier based SVM is as follows:

  Level 1: Set up image type sets.
  Level 2: Generate functional Bag.
  Level 3: Training the image with BoVwords.
  Level 4: Classification using SVM classifier.

Based on the operation of the BOV classifier, the images are processed for examination, specifically, the image is divided into two parts: (1) training and (2) testing subjects. After that, the takeout support vector machine produces a visual vocabulary from each package's representative images. The image is extracted from the training set in the process used to extract the characteristics from the image. Using the nearest neighbor algorithm, an image histogram function is constructed. The histogram converts the image into a function vector. Classification finally is done with SVM classifier assistance.

#### 2.6.3. Convolutional Neural Network

Deep learning methodology is used for arranging the information mainly into four objective factors and to check its precision for each point. Very few investigations were conveyed utilizing different classifications from this informative collection. Deep learning is a kind of AI that manages calculations roused by brain structure and capacity, called neural artificial networks. The thing that isolates it from neural systems is the huge realizing, which is utilized to explain the advancement of new technology in an ANN to process bigger measures of information and to improve its precision of the data classification [36]. Convolution Neural Network (CNN) is an exceptional sort of neural system for preparing information in image, text, and sound structures that have worked effectively in their usage [25]. The expression “Convolution Neural Network” built up a measurable activity called convolution, to show their network. The convolution operation is the operation of a dot product between the process's input matrices. The working of the CNN is presented in Figure 6, and the basic architecture is presented in Figure 7.

Convolutional Neural Network relies upon connecting the previous layer's local territory to the following layer. Spatially, CNN sets up a neighborhood relationship by applying a progressive example of communication between neurons of adjoining layers. The one-layer units connect to the former layer subunits. Preceding layer unit number forms map width. The subsequent rendition takes motivation from the Lanet-5. This standard of forcing neighborhood, availability is portrayed, as observed in Figure 8.

Anyway, as in customary multilayer systems, CNN shares loads; the measure of accessible boundaries does not expand considerably to the input measurements. The main elements of CNN-2 layer classifiers are explained below:

*(1) The Convolutional Layer*. Behaviors of a 2D sifting between *x*-input images and *w* channel bank, producing an extra assortment of *h* images. Input-output correspondences are shown by an association table; channel reactions are consolidated straightly from the input associated with a similar output image. An association with the accompanying semiconductor is framed through the MRI column: (input Image, separated, output Image). This layer does the mapping after

(13) $$\begin{array}{c} h_{j}=\sum_{i,k\in CT_{i,k,j}}x_{i}*w_{k}, \end{array}$$

where ^*∗*^ shows true 2D convolution. A given layer's *w*_*k*_ the channel has a similar size, and *x*_*i*_ determines the size of the output image alongside the input value *h*_*j*_. Likewise with standard multilayer systems, ‘he is then applied to the nonlinear activation function.

*(2) Pooling Layer*. The pooling layer does not mean to lessen the calculation unpredictability, however, in addition to the direct decision of the feature. The input images are tiled in uncorrelated subareas, which recover just one output an incentive from. Most extreme or normal mainstream choices, ordinarily named as max-pooling and avg-pooling. The max-pooling is normally profitable given that it adds a slight invariance to interpretation and distortion, which in turn prompts quicker assembly and better speculation.

*(3) Fully Connected Layer*. In the layered system, a fully connected layer acts as a base layer. Either the system switches convolutional and max-pooling layers with the 1D feature vector the gotten at some stage, or the outcomes collected are redesigned for 1D structure. The base layer is directly connected to the classification process, with the same number of neurons as classes. With a softmax activation function, the outputs are normalized, and in this way gauge probabilities of the back class. Various measuring techniques such as size and number of capabilities maps bit sizes, factor skipping, and connection table are used in the convolution layer.

In the proposed system, the bit size utilized by the connected layer is 7 × 7, the number of feature maps compared to 6 for the main layer of convolution, and the second layer of convolution equivalent to 12. The skipping component in the network decides the horizontal and vertical pixel number by which the part will skip between ensuing convolutions. In each layer where *M* includes the size maps (*M*_*x*_, *M*_*y*_), the size part (*K*_*x*_, *K*_*y*_), the skipping factors (*S*_*x*_, *S*_*y*_) are than the size relationship of the output maps as per the above parameters:

(14) $$\begin{array}{c} Mnx=M_{n-1x}-k_{nx}S_{nx}+1,\\ Mny=M_{n-1y}-k_{ny}S_{ny}+1, \end{array}$$

where the layer is demonstrated by the record “*n*.” In layer *Ln* − 1 at most, each map in layer *Ln* is associated with *Mn*−1 maps. Neurons of a given map share their loads yet have distinctive open fields.

The information layer has a component map compared to the size of the character's standardized image. In this exploration, masses are arbitrarily picked from a uniform dispersion inside the range [−1/fan-in, 1/fan-in] where the contributions to a hidden variable are given by fan-in. For CNN, this relies upon the quantity of feature maps input and the size of the open field. Likewise, with the CNN case, max-pooling is a nondirect down-example. The input image is partitioned into a collection of nonoverlapping rectangles by methods for max-pooling, and yields are determined as the most elevated advantage for each such sublocale [26].

For two reasons, max-pooling is useful in vision:

- reduces the numerical sophistication of the upper strata.
- It provides different types of invariance in translation.

The second layer of convolution layer comprises six component maps which are gotten by interpreting the size 5 × 5 pieces into the feature map of the info. The subtesting layer is shown in the third layer, and it is employed in the downexamining of the image. For a downsampling of the image, the max-pooling method is employed over the 2 × 2 region of the input image. The convolution layer, which is the third layer, makes the changes over the image to a partition size of 5 × 5 based on the feedback from the past layer. At this stage, the number of feature maps acquired equivalents 12. Again, the subinspecting is acted in the fourth layer with the procedure max-pooling in the area of size 4 × 4. The fifth layer is a fully associated layer that drives a classifier to give a feedforward yield.

The training part considers the elements in layers 1–4 are the extraction part of the trainable element, and the classifier is the following replacement layer. Images are partitioned into a test set and preparing the set. Every computerized image was size-standardized and dependent on a 28 × 28-pixel fixed-scale image. In the first dataset, each pixel of the image is portrayed by an incentive somewhere within the range of 0 and 255, where 0 is dark, 255 is white, and everything in the middle is an alternate shade of dim. An image is represented as a 1-dimensional array of float esteems of 784 (28 × 28) from 0 to 1 (0 methods dark, 1 method white). At the point when we utilize the dataset, we split the preparation and test cluster into smaller than normal bunches.

#### 2.6.4. Performance Analysis

The following performance metrics are obtained from the segmentation and classified result.

Detection part:

(15) $$\begin{array}{c} \text{Jaccard index}=J\left(A,B\right)=\;\frac{S\left(A\cap^{}B\right)}{S\left(A\cup^{}B\right)}.\\ \text{Dice overlap index}\left(\text{DOI}\right)=D\left(A,B\right)=2X\frac{A\cap^{}B}{A+B},\\ \text{Similarity index SI}=\frac{2X\text{Truepositive}}{2X\text{truepositive}+\text{falsepositive}+\text{falsenegative}},\\ \text{Absolute volume measurement error}\left(AVME\right)=\left(\frac{V_{automatic}}{V_{manual}}-1\right)\times 100\%,\\ \text{Figure of merit}\left(\varepsilon \right)=1-\left(\varepsilon \right)=1-\frac{\left|V_{\text{manual}}-V_{\text{automatic}}\right|\;}{V_{\text{manual}}}. \end{array}$$

Classification part:

(16) $$\begin{array}{c} \text{Sensitivity}=\frac{TP}{TP+FN}\times 100\%,\\ \text{Specificity}=\frac{TN}{TN+FP}\times 100\%,\\ \text{Accuracy}=\frac{TP+TN}{TP+FP+FN+TN}\times 100\%. \end{array}$$

## 3. Results and Discussion

The suggested strategy was created using MATLAB software that has a Core 2 Duo code configuration. Initially, the preprocessing technique is applied to enhance the image. Next, the segmentation is applied to extract the boundary region of the tumor. The result is shown in Figures 9 and 10.

In our approach after applying the fitness function of the GA, the optimized features considered are mean, variance, skewness, kurtosis, and energy. The result is shown in Table 1. The cycle of classification is divided into two parts (i.e., the training part and the evaluation part). First, known data (i.e., 24 features^*∗*^ 46 images) are given in the training part to the training classifier. Second, unknown data are provided to the classifier in the testing phase, and the classification is carried out after the training part. The classification's accuracy rate and error rate depend on the quality of the training.

Figures 11–13show the results of GA, and Figure 14 shows the visual word occurrence of the BoVW classifier. Here, the *x*-axis represents the visual word index, and the *y*-axis represents the frequency of occurrences in the images correspondingly. The obtained accuracy and confusion matrix is shown in Figures 15 and 16. The obtained accuracy of the proposed classifier is 90% and 97.3%. Table 1 shows the performance value of the suggested classifier.  Table 2 presents the statistical analysis of the brain images, and Table 3 presents the performance comparisons.

Further, the findings have acquired an average index coefficient of 0.82 dice similarity, suggesting a greater comparison between the computerized tumor areas (machines) extracted by radiologists and manual tumour region extraction Our current technique results demonstrated the importance of quality parameters and accuracy compared to state-of-the-art techniques.

In CNN, the model ResNet-50 consists of 5 stages, each with a convolution block and identity block. Each block of convolution has three layers, and every block of identity has three layers of convolution too. The ResNet-50 has more than 23 million trainable parameters. Figures 17 and 18 show the first line of ResNet and First Convolution Layer Weights. A confusion matrix is a table that is sometimes used to explain the output of a classification model over a set of test data defined for true values. It enables the output of an algorithm to be visualized. In a projected class, the matrix row represents instances, while each column represents instances in a real class (or vice versa).  Figure 19 shows the matrices obtained for precision and uncertainty. The accuracy obtained is 98.5 percent. Figures 20 and 21 show the plot of different classifiers for performance.

## 4. Conclusion

Medical image segmentation is a challenging issue due to the complexity of the images, as well as the lack of anatomical models that fully capture the potential deformations in each structure. This proposed method works very effectively to the initial cluster size and cluster centers. The segmentation is done by using BWT techniques whose accuracy and computation speed are less. This work recommends a system that requires negligible human intrusion to partition the brain tissue. The main aim of this recommended system is to aid the human experts or neurosurgeons in identifying the patients with minimal time. The experimental results show 98.5% accuracy compared to the state-of-the-art technologies. Computational time, system complexity, and memory space requirements taken for executing the algorithms could be further reduced. The same approach can be also used to detect and analyze different pathologies found in other parts of the body (kidney, liver, lungs, etc.). Different classifiers with optimization methodology can be used in future research to improve accuracy by integrating more effective segmentation and extraction techniques with real-time images and clinical cases using a wider data set covering various scenarios.

## Figures and Tables

**Figure 1:** Basic block diagram of planned work.

**Figure 2:** Features selected for CNN techniques.

**Figure 3:** GA-based feature selection.

**Figure 4:** Matrix representation showing the bit value of chromosome in genetic algorithm.

**Figure 5:** Block diagram showing the steps for support vector machine training and testing.

**Figure 6:** Basic diagram for the working of CNN.

**Figure 7:** The Convolutional Neural Network basic architecture.

**Figure 8:** Local connections pattern representation.

**Figure 9:** Preprocessing results.

**Figure 10:** Result of the proposed segmentation in FLAIR and T2 images.

**Figure 11:** Feature selection result using GA.

**Figure 12:** Fitness function using GA.

**Figure 13:** Crossover and mutation result.

**Figure 14:** Visual word occurrence of the BoVW.

**Figure 15:** Confusion matrix of Naïve Bayes.

**Figure 16:** Confusion matrix of BOVW based SVM classifier.

**Figure 17:** First section of ResNet.

**Figure 18:** First convolution layer weights.

**Figure 19:** The confusion matrix of proposed CNN.

**Figure 20:** Accuracy and error plot.

**Figure 21:** Accuracy, sensitivity, and precision plot.

**Algorithm 1:** Algorithm for genetic algorithm.

**Table 1:** Optimized feature extracted after applying genetic algorithm.

Image no.	First-order statistics (FOS) feature				
	Mean	Standard deviation	Skewness	Kurtosis	Entropy
1	0.011	0.019105	2.274177	7.10785	2.68715
2	0.006	0.010301	1.605176	4.28244	2.05357
3	0.008	0.010716	1.578003	4.13867	2.57759
4	0.010	0.01203	0.826578	2.47775	2.77483
5	0.011	0.01429	0.945757	2.65592	2.23901
6	0.010	0.008143	0.419944	2.28365	2.81441
7	0.014	0.01945	2.495946	12.0050	3.11189
8	0.012	0.01388	1.159288	3.16243	3.16398
9	0.014	0.02124	2.216729	9.24762	2.65219
10	0.008	0.010971	1.308686	4.27185	2.4252

**Table 2:** Statistical analysis of the brain images.

Image	Dice coefficient	Jaccard's coefficient	Spatial overlap	AVI	Spatial overlap	VOI of segmented ROI	Accuracy	Specificity	Time elapsed	Figure of merit
1	0.85	0.81	0.891	24.349	0.892	859	98.58	99.5838	0.687	0.826
2	0.89	0.79	0.833	−28.549	0.834	532	98.91	99.6829	0.7011	0.799
3	0.87	0.88	0.912	−19.46	0.97	577	98.88	99.6765	0.6835	0.978
4	0.79	0.81	0.888	−22.163	0.884	723	99.02	99.6969	0.6524	0.787
5	0.73	0.89	0.967	−7.889	0.961	785	99.18	99.8522	0.9601	0.232
6	0.85	0.82	0.878	29.862	0.875	935	99.16	99.8343	0.980	0.612
7	0.87	0.88	0.914	20.134	0.917	925	99.11	99.7590	0.7404	0.939
8	0.89	0.71	0.762	−39.225	0.768	444	99.06	99.8163	0.8194	0.967
9	0.85	0.89	0.938	−13.315	0.939	794	98.88	99.5867	0.677	0.653
10	0.87	0.88	0.913	−16.892	0.913	775	98.73	99.7162	0.699	0.477

**Table 3:** Performance comparison.

Classifier	Naïve Bayes (%)	BoVW-based SVM (%)	CNN (%)
Accuracy	90	97.3	98.5
Error	10	2.7	1.5
Sensitivity	86.6	98.6	98.6
Specificity	84	96.1	97
Precision	93.3	96	98

## Data Availability

Data will be available from the corresponding author upon request.
